The article "Efficacy of Ambroxol Hydrochloride Combined with Amoxicillin Potassium Clavulanate Combination on Children with Bronchopneumonia and Its Impact on the Level of Inflammatory Factors" was retracted in 2023. Reasons: unreliable results or conclusions; concerns about the data; concerns about the peer review; concerns about the citations.

# Efficacy of Ambroxol Hydrochloride Combined with Amoxicillin Potassium Clavulanate Combination on Children with Bronchopneumonia and Its Impact on the Level of Inflammatory Factors

**DOI:** 10.1155/2022/2604114

**Published:** 2022-08-19

**Authors:** Xiaoli Zhu, Zongcheng Wei, Xia Liu

**Affiliations:** ^1^Nanjing Pukou District Hospital of Traditional Chinese Medicine, Pediatric Department, Nanjing, China; ^2^Nanjing Pukou District Hospital of Traditional Chinese Medicine, Equipment Section, Nanjing, China

## Abstract

**Objective:**

The goal of the present study was to examine the effect of ambroxol hydrochloride combined with amoxicillin potassium clavulanate combination on children with bronchopneumonia and its influence on the level of inflammatory factors.

**Methods:**

From January 2018 to June 2019, 100 children with bronchopneumonia admitted to the Pediatric Department of Nanjing Pukou District Hospital of Traditional Chinese Medicine were enrolled as the study subjects. The children were assigned either to an observation group or a control group in a ratio of 1:1 using the random alphabet method. The observation group was treated with ambroxol hydrochloride plus amoxicillin potassium clavulanate combination, and the control group was treated with amoxicillin potassium clavulanate combination. The therapeutic efficiency and serum white blood cells (WBC), C-reactive protein (CRP), interleukin-6 (IL-6), and tumor necrosis factor-a (TNF-*α*) were compared between the two groups.

**Results:**

Regarding the effective rate of treatment, the observation group (94%) was observed to be notably higher as compared to the control group (84%). The levels of WBC, CRP, IL-6, and TNF-*α* were reported to be significantly lower in the two groups after treatment. The WBC, CRP, IL-6, and TNF-*α* after treatment in the observation group were lower than those in the control group. The time for clinical symptoms to disappear of fever, cough, asthma, and pulmonary rales was all shorter in the observation group.

**Conclusion:**

The findings of the present study demonstrate that ambroxol hydrochloride combined with amoxicillin potassium clavulanate combination might be a reliable approach for the treatment of bronchopneumonia in children. It can synergistically relieve inflammation with high safety profiles.

## 1. Introduction

Bronchopneumonia, also known as lobular pneumonia, is one of the most common infant infectious diseases that leads them to be hospitalized. The contributing factors are one or multiple pathogenic microorganism infections of bacteria, viruses, and mycoplasma *pneumoniae*, and the main clinical signs and symptoms include fever, cough, asthma, vomiting, irritability, dyspnea, and pulmonary rales [1]. The mainstays of bronchopneumonia include inflammation control, ventilation improvement, prevention, and treatment of complications. [2]. Bronchopneumonia belongs to the category of “pneumonia and cough” in traditional Chinese medicine (TCM). The main clinical manifestations are fever, cough, wheezing, and nasal fans. The incidence rate of bronchopneumonia in children is high because of the stenosis of the trachea and bronchial lumen, the lack of mucus secretion, the occurrence of mucus blockage, and the incomplete development of the overall respiratory system [3]. However, for reasons such as children's compliance, TCM decoction is rarely used.

Ambroxol hydrochloride is one expectorant for treating respiratory system diseases related to abnormal mucous secretion and damaged mucous transport by promoting mucous clearance and sputum excretion, relieving cough, and controlling inflammation. The use of ambroxol hydrochloride is deemed effective to restore the physiological clearance mechanism of the respiratory tract via stimulating the synthesis and release of the surface reactive substance and decreasing mucus's adherence to the bronchial wall [4]. Ambroxol is an antioxidant mucus-dissolver that plays an important role in protecting infants' respiratory systems. Amoxicillin potassium clavulanate combination is an antisepsis and anti-inflammation medicine made from amoxicillin potassium clavulanate combination disproportionately. It is a reliable strategy for treating lower respiratory tract infections, otitis media, nasosinusitis, urinary tract infections, skin, soft tissue infections, and other diseases [5].

Currently, both drugs have been applied to the treatment of bronchitis pneumonia in children [6, 7]. However, there are few studies on the combined application. In this regard, this study aims to investigate the effect of ambroxol hydrochloride combined with amoxicillin potassium clavulanate combination on children with bronchial pneumonia and its impact on the level of inflammatory factors.

## 2. Materials and Methods

### 2.1. General Information

From January 2018 to June 2019, 100 children with bronchopneumonia admitted to the Pediatric Department of Nanjing Pukou District Hospital of Traditional Chinese Medicine were enrolled as the study subjects. The children were assigned either to an observation group or a control group in a ratio of 1 : 1 using the random alphabet method. The study has been reviewed and approved by the medical ethics committee (no. 2018/14–524), and the family members of the children provided informed consent prior to its commencement.

### 2.2. Inclusion and Exclusion Criteria

#### 2.2.1. Inclusion Criteria

(1) patients who met the diagnostic criteria for bronchial pneumonia [8]; (2) children who had not received antibiotic therapy 24 hours prior to admission; (3) children who had no serious systemic disease and injury of the liver and the kidney; (4) children who had no history of drug allergy.

#### 2.2.2. Exclusion Criteria

(1) children with severe respiratory and circulative system diseases; (2) children with unclear pathogenesis; (3) children with pulmonary infections or other severe diseases; (4) children with drug allergies.

### 2.3. Treatments

Both groups were given conventional symptomatic treatment upon admission, including relieving cough, oxygen inhalation, reducing phlegm, and fever reduction. On this basis, the control group was given an intravenous injection of amoxicillin potassium clavulanate combination (North China Pharmaceutical Co. Ltd, SFDA approval number: H20054213) at a dose of 50 mg/kg per time, once every 8 hours. The observation group was given an additional intravenous injection of ambroxol hydrochloride (AstraZeneca Pharmaceutical Co. Ltd, SFDA approval number: H20120906) at a dose of 30 mg/kg per time, once every 8 hours. One week was taken as a course of treatment. Medication should be stopped in the case of any severe adverse reactions. If there is no pronounced efficacy after the first course of treatment, another course or other medication should be given.

### 2.4. Therapeutic Effect Criteria

The therapeutic effects are categorized into (1) cured: patients' signs and symptoms disappeared after a course of treatment with a clear lung image using chest X-ray; (2) effective: patients' signs and symptoms significantly mitigated with marked reduction of lung shadows using chest X-ray; (3) ineffective: no significant improvement or even aggravation in signs and symptoms was observed with no reduction or increase of lung shadows using chest X-ray. Effective rate = (Cured + Effective)/Total cases × 100%.

### 2.5. Outcomes

During the treatment, the signs and symptoms of all pediatric patients were monitored, and the disappearance time of fever, cough, asthma, and pulmonary rales was recorded. 5 ml of venous blood was collected before and after the treatment and centrifuged, and then, the serum was secured. The white blood cell (WBC) count was evaluated by an automatic hematology analyzer (SYSMEX-5000). The serum level of C-reactive protein (CRP) was evaluated by immunoturbidimetry (Cobas E 801). The serum levels of interleukin-6 (IL-6) and tumor necrosis factor-a (TNF-*α*) were evaluated by enzyme-linked immune sorbent assay (ELISA) kits. The kit of IL-6 was provided by Abcam (cat no. ab178013); the kit of TNF-*α* was provided by Elabscience (cat no. E-EL-H0109c).

### 2.6. Statistical Analysis

The statistical analysis was conducted using SPSS Statistics software 22.0. All measurement data were tested for normality first, and those that did not conform to normal distribution were transformed for normality. The enumeration data were represented by (*n* (%)) and analyzed by the chi-square test. The measurement data were represented by $\left(\bar{x}\pm s\right)$ and analyzed by the *t*-test. Significance was claimed at a *p* value of less than 0.05.

## 3. Results

### 3.1. General Information

The children aged 2–6 years old, with the average of 4.41 ± 0.72 years and the average course of 7.89 ± 3.44 days. The differences did not reach statistical significance in the baseline data (*p* > 0.05, Table 1).

### 3.2. Therapeutic Efficiency

31 cases were cured in the observation group, and 21 cases were cured in the control group. The effective rate in the observation group was higher than the control group (94.00% vs. 84.00%) (*p* < 0.05, Table 2).

### 3.3. WBC Count

Prior to treatment, the WBC of the observation group and the control group were, respectively, 16.75 × 109/L and 16.54 × 109/L, which were not significantly different (*p* > 0.05). Both groups witnessed a marked decrease in the WBC after treatment, with the observation group having a lower value than the control group ((5.13 × 109/L) vs. (9.69 × 109/L)) (*p* < 0.05, Figure 1).

### 3.4. Inflammatory Factors

No differences were observed in the serum in terms of the level of CRP, IL-6, and TNF-*α* between the two groups prior to treatment; all the parameters significantly decreased after treatment (*p* < 0.05), with greater reduction observed in the observation group compared to the control group (*p* < 0.05, Table 3).

### 3.5. Time for Clinical Symptoms to Disappear

The time for clinical symptoms to disappear for fever, cough, asthma, and pulmonary rales were all shorter in the observation group compared to the control group (*p* < 0.05, Table 4).

### 3.6. Adverse Reaction

The two groups had a similar safety profile with no noticeable adverse reaction in the two groups.

## 4. Discussion

Due to the fact that infants and children's immune systems have not fully developed, they are prone to suffering bronchopneumonia caused by infections from bacteria, viruses, and other pathogens [9]. At the moment, penicillin is the main medication for bronchopneumonia in children, but it is associated with resistance to pathogenic microorganisms, which hinders its the clinical efficacy [10].

This study found that the effective rate of treatment of ambroxol hydrochloride plus amoxicillin potassium clavulanate combination is significantly higher than that of amoxicillin potassium clavulanate combination. Amoxicillin is a widely used semisynthetic penicillin's broad-spectrum *β*-lactam antibiotic, which has strong absorbability and can sterilize and permeate cell membranes in the gastrointestinal tract. Although it has low antimicrobial activity, clavulanate potassium binds to the majority of enzymes within the *β*-lactam and inhibits their activity [11]. Therefore, clavulanate potassium combined with penicillins has favorable clinical efficacy in inflammatory infectious diseases [12]. The interpretation can be attributed to the fact that ambroxol hydrochloride reduces the inflammatory responses by promoting sputum excretion and clearing pathogenic bacteria; thus, it can relieve cough and other symptoms. Amoxicillin potassium clavulanate combination can counter the drug resistance of pathogenic bacteria. As a result, a promisingly synergistic effect was produced using ambroxol hydrochloride combined with amoxicillin potassium clavulanate combination.

In this study, the WBC, CRP, IL-6, and TNF-*α* after treatment in the observation group were lower than those in the control group. Leukocytes are blood cells that can phagocytose foreign bodies and produce antibodies, which are closely related to the body's immunity and resistance to pathogens. In clinical practice, WBC is often considered an indicator of infection, inflammation, physical trauma, and disease progression [13]. CRP is a common indicator of inflammation caused by bacterial infection and has a high sensitivity to acute infection. IL-6 is an interleukin encoded by the gene IL6. IL-6 is secreted by T cells and macrophages, stimulates immune responses, and plays an important role in infection and tissue damage [14]. TNF-*α* is a cell signaling protein involved in systemic inflammatory response; it is produced by the activation of macrophages, neutrophils, lymphocytes, and other cells, and it is one of the cytokines in acute inflammatory phase infection [15]. According to the results, children with bronchitis and pneumonia have a higher level of WBC and higher expression of inflammatory factors such as CRP, IL-6, and TNF-*α*. After the proper treatment, the four indicators have significantly decreased [16, 17]. Moreover, the treatment with ambroxol hydrochloride combined with amoxicillin potassium clavulanate combination resulted in lower WBC and inflammatory factors as compared with amoxicillin potassium clavulanate combination, suggesting a prominent efficacy of ambroxol hydrochloride combined with amoxicillin potassium clavulanate combination in the treatment of bronchitis pneumonia in children. The possible explanation may be that the drug combination can promote the removal and sterilization of pathogenic bacteria, thereby reducing the inflammatory response and exerting a therapeutic effect [18, 19]. Importantly, no noticeable adverse reactions were found, suggesting a satisfactory safety profile.

However, this study still has the following limitations. First of all, the follow-up time of this study was short. The efficacy and various indicators were compared only one week after treatment, so the long-term efficacy and safety evaluation were insufficient. Secondly, the sample size of this study was small, with only 50 patients in each group, and the reliability of evidence was insufficient. At the same time, children's compliance is poor, and the treatment effect is also affected by family, nursing, and other factors, so the heterogeneity is difficult to exclude.

## 5. Conclusion

Ambroxol hydrochloride plus amoxicillin potassium clavulanate combination is effective in the treatment of bronchopneumonia with acceptable safety. It, therefore, warrants a promotion in clinics.

## Figures and Tables

**Figure 1:** WBC in two groups of children with bronchopneumonia before and after treatment. Note: BT: before treatment; AT: after treatment; OG: observation group; CG: control group; ^*∗*^: compared with BT, *p* < 0.05; ^#^: compared with OG, *p* < 0.05.

**Table 1:** General information.

Data	Observation group (*n* = 50)	Control group (*n* = 50)	*χ* ^2/*t*^	*p*
Gender (*n*)			0.161	0.688
Male	28	26		
Female	22	24		
Age (year)	4.13 ± 0.85	4.81 ± 0.74	2.433	0.478
Course of disease (d)	7.48 ± 3.35	8.29 ± 3.50	1.426	0.519

**Table 2:** Therapeutic effects.

Group	Cured	Effective	Ineffective	Effective rate (%)
Observation group (*n* = 50)	31	16	3	94.00
Control group (*n* = 50)	21	21	8	84.00
*χ* ^2^			2.167	
*p*			0.030	

**Table 3:** Serum CRP, IL-6, and TNF-*α.*

Group	CRP (mg/L)		IL-6 (ng/L)		TNF-*α* (ng/L)	
	Before	After	Before	After	Before	After
Observation group (*n* = 50)	33.35 ± 6.27	31.53 ± 4.38	3.03 ± 0.89	2.91 ± 0.92	7.68 ± 1.26	8.03 ± 1.36
Control group (*n* = 50)	2.36 ± 1.17	8.25 ± 3.46	0.67 ± 0.12	1.59 ± 0.10	3.11 ± 0.56	4.52 ± 0.79
*t*	54.765	47.854	11.647	1.745	13.754	5.769
*p*	<0.001	<0.001	0.001	0.005	0.001	0.011

**Table 4:** Time for clinical symptoms to disappear.

Group	Fever	Cough	Asthma	Pulmonary rales
Observation group (*n* = 50)	2.32 ± 0.54	4.25 ± 0.84	3.21 ± 0.51	4.02 ± 0.95
Control group (*n* = 50)	3.14 ± 0.61	5.84 ± 0.75	4.17 ± 0.62	5.11 ± 1.04
*t*	7.117	9.984	8.456	5.472
*p*	<0.001	<0.001	<0.001	<0.001

## Data Availability

The datasets used during the present study are available from the corresponding author upon reasonable request. All data generated or analysed during this study are included within this published article.

## References

[1] Britton A. P., Redford T., Zabek E. (2017). Bronchopneumonia associated with Mannheimia granulomatis infection in a Belgian hare (Lepus europaeus). *Journal of Veterinary Diagnostic Investigation*.

[2] Elfadl A. K., Lee S. W., Kim J. H. (2017). Fatal fibrino-hemorrhagic bronchopneumonia associated with *Morganella morganii* in a bottlenose dolphin: a case report. *Diseases of Aquatic Organisms*.

[3] Shang X., Liabsuetrakul T., Sangsupawanich P., Xia X., He P., Cao H. (2015). Satisfaction and preference for traditional Chinese medicine drugs among guardians of children with acute bronchiolitis. *Journal of Alternative & Complementary Medicine*.

[4] Yang Z., Xiao X., Huang Y. (2017). Effects and mechanisms of ambroxol inhalation (MucosolvanⓇ) in the treatment of neonatal pneumonia. *Pharmazie*.

[5] Marra M. C., Cunha R. R., Muñoz R. A. A., Batista A. D., Richter E. M. (2017). Single-run capillary electrophoresis method for the fast simultaneous determination of amoxicillin, clavulanate, and potassium. *Journal of Separation Science*.

[6] Liu H., Wang W., Gao X. (2020). Comparison of the efficacy of ambroxol hydrochloride and N -acetylcysteine in the treatment of children with bronchopneumonia and their influence on prognosis. *Experimental and Therapeutic Medicine*.

[7] Mihani J., Këlliçi S. (2018). Patterns of antibiotic prescription in children: tirana, Albania region. *Open Access Macedonian Journal of Medical Sciences*.

[8] Asano K., Hebisawa A., Ishiguro T. (2021). New clinical diagnostic criteria for allergic bronchopulmonary aspergillosis/mycosis and its validation. *The Journal of Allergy and Clinical Immunology*.

[9] Murray G. M., More S. J., Sammin D. (2017). Pathogens, patterns of pneumonia, and epidemiologic risk factors associated with respiratory disease in recently weaned cattle in Ireland. *Journal of Veterinary Diagnostic Investigation*.

[10] Rutenberg D., Venner M., Giguère S. (2017). Efficacy of tulathromycin for the treatment of foals with mild to moderate bronchopneumonia. *Journal of Veterinary Internal Medicine*.

[11] Sood S., Gupta V. K., Agarwal S., Dev K., Pathania D. (2017). Controlled release of antibiotic amoxicillin drug using carboxymethyl cellulose-cl-poly (lactic acid-co-itaconic acid) hydrogel. *International Journal of Biological Macromolecules*.

[12] Leung A. K. C., Wong A. H. C., Leung A. A. M., Hon K. L. (2019). Urinary tract infection in children. *Recent Patents on Inflammation & Allergy Drug Discovery*.

[13] Wan B., Zhang H., Fu H. (2015). Recombinant human interleukin-11 (IL-11) is a protective factor in severe sepsis with thrombocytopenia: a case-control study. *Cytokine*.

[14] Pournot H., Bieuzen F., Louis J. (2011). Time-course of changes in inflammatory response after whole-body cryotherapy multi exposures following severe exercise. *PLoS One*.

[15] He S., Wang L., Miao L. (2009). Receptor interacting protein kinase-3 determines cellular necrotic response to TNF-*α*. *Cell*.

[16] Cheng Q., Zhang H., Shang Y. (2021). Clinical features and risk factors analysis of bronchitis obliterans due to refractory Mycoplasma pneumoniae pneumonia in children: a nomogram prediction model. *BMC Infectious Diseases*.

[17] Pan C., Chen Y., Wang S., Li M., Qu S. (2021). The study of routine laboratory factors in children with mycoplasma pneumoniae pneumonia: serum uric acid may have anti-inflammatory effect. *Journal of Clinical Laboratory Analysis*.

[18] Wang F., Nan K., Hao L. (2021). Effects of a combination of erythromycin sequential therapy and azithromycin on lung function and inflammatory factors in children with severe mycoplasma pneumonia. *Pakistan Journal of Pharmaceutical Sciences*.

[19] Yin M. (2021). Effect of Qingfei Huatan Huoxue Decoction combined with azithromycin on pulmonary function and inflammatory factors in children with Mycoplasma pneumonia. *Pakistan journal of Pharmaceutical Sciences*.

